# The relationship between spiritual well-being and fear of cancer progression in Iranian cancer patients

**DOI:** 10.3389/fpsyg.2025.1495988

**Published:** 2025-01-22

**Authors:** Amir Hossein Goudarzian, Seyed Amirhossein Mazhari, Pooria Sobhanian, Bahar Farhadi, Soheyla Kalantari, Mozhgan Taebi

**Affiliations:** ^1^Department of Psychiatric Nursing, School of Nursing and Midwifery, Tehran University of Medical Science, Tehran, Iran; ^2^Student Research Committee, Mazandaran University of Medical Sciences, Sari, Iran; ^3^Student Research Committee, Azerbaijan Medical University, Baku, Azerbaijan; ^4^Student Research Committee, Faculty of Medicine, Mazandaran University of Medical Sciences, Sari, Iran; ^5^School of Medicine, Islamic Azad University, Mashhad, Iran; ^6^Laboratory Science Research Center, Surgical Technology Department, Golestan University of Medical Sciences, Gorgan, Iran; ^7^Department of Anesthesiology, Faculty of Allied Medical Sciences, Kerman University of Medical Sciences, Kerman, Iran

**Keywords:** spiritual well-being, fear of cancer progression, cancer, Iran, oncology

## Abstract

**Introduction:**

This study aimed to investigate the nuanced relationship between spiritual well-being and fear of cancer progression among individuals diagnosed with cancer.

**Methods:**

The study was conducted in 2023 and utilized a predictive cross-sectional survey. A total of 398 cancer patients were recruited using convenience sampling. The Spiritual Well-Being Scale (SWBS) and the Fear of Progression (FOP) scale were used for data collection. Data analysis was performed using SPSS version 26, AMOS, and JASP to assess the reliability of the constructs and the potential relationship between the two main variables.

**Results:**

The mean age of the participants was 49.14 years (SD = 16.16, 95% CI: 47.55 50.74). All constructs demonstrated strong factorial validity and reliability. Simple linear regression analysis revealed that spiritual well-being significantly predicted fear of cancer progression (*R*^2^ = 0.064, *F* = 27, *p* < 0.001).

**Discussion:**

The findings indicated a significant relationship between spiritual well-being and fear of cancer progression. These results highlighted the interconnectedness of spiritual well-being and fear of cancer progression among cancer patients.

## Introduction

Cancer is a major global health issue, causing millions of deaths each year and significant morbidity (Pinto et al., 2022). In 2020, over 10 million people worldwide died from cancer (Sung et al., 2021). In Iran, 131,191 new cases of cancer and 79, 136 cancer-related deaths were reported in 2020. Among these cases, breast cancer was the most frequently diagnosed type (12.9%), followed by stomach (11.2%), colorectal (9.1%), lung (8%), and prostate (6.8%) cancers (Ferlay et al., 2020). A study predicts a 40% increase in new cancer cases in Iran by 2025, highlighting the growing burden of cancer in the country (Roshandel et al., 2021).

Receiving a cancer diagnosis can be emotionally challenging for individuals due to the fear of an incurable disease and shortened life expectancy. This can lead to significant psychological and physical distress, affecting their overall quality of life, which is an important measure of health (Shrestha et al., 2019; Turchi et al., 2022).

Fear of cancer progression (FCP) is a common and complex emotional response among cancer patients. It stems from the uncertainty of the disease and the fear of its advancement despite ongoing treatment (Bergerot et al., 2022). Patients struggle with the physical and emotional toll of living with the constant uncertainty of their future (Coutts-Bain et al., 2022). As treatment continues, this fear may shift to concerns about treatment side effects, changes in quality of life, or the need for more aggressive interventions (Dinkel and Herschbach, 2018).

The fear of cancer recurrence, known as FCP, can linger for years following treatment, fueled by uncertainty about the unpredictable nature of the disease (Bergerot et al., 2022). Patients face ongoing concerns about their health, symptoms, and the impact of cancer on their daily lives. This persistent uncertainty can worsen FCP, leading to a cycle of anxiety and distress. Managing FCP is essential for mental well-being, treatment compliance, and overall prognosis (Ocalewski et al., 2021).

Psychosocial factors, such as spiritual mechanisms, social support networks, and individual resilience, are crucial in influencing the intensity and expression of FCP (Nahm et al., 2021; Yang et al., 2018). Patients may feel increased anxiety when they believe they have little control over their situation, grapple with existential issues, or find it difficult to communicate their fears to healthcare providers, family, and friends (Nahm et al., 2021). Spirituality, which is often described as a deeply personal connection to a higher power, can provide significant comfort and support for individuals facing the challenges of a cancer diagnosis (Ali et al., 2023).

One important aspect that could influence the management of FCP is spiritual well-being. Spirituality can offer individuals a sense of significance, tranquility, and direction, which is especially crucial when dealing with serious illnesses like cancer. In various societies, such as in Iranian culture, spirituality is an integral part of everyday life and can serve as a significant source of solace and resilience (Ahmadi et al., 2021).

There is a very strong association between spiritual well-being and psychological health, particularly in patients facing fatal diseases like cancer. Theoretically, the basis for such an association between spiritual well-being and psychological health is: giving meaning, lessening mortality anxiety, and thereby generating an inner feeling of peace (Liu et al., 2022). In cancer patients, these existential questions-thoughts about life and death-increase psychological distress. Spiritual well-being attends to such concerns by offering a means in which one interprets this experience and ascribes meaning and purpose to the suffering (Ellington et al., 2017). Often, spiritual experiences reinterpret suffering as an opportunity for growth and resilience. Spiritual well-being may help mitigate FCP as it reduces anxiety about dying and promotes acceptance. Through mindfulness and prayer, people feel connected to something greater than themselves-a higher power or community-and come to a state of serenity and self-control in the presence of uncertainty (Zhang et al., 2022). It also forms the theoretical framework for investigating the relation of spiritual well-being and FCP among participants for whom spirituality is both personally and communally significant, in their cultural contexts (Zhang et al., 2022).

For many cancer patients, dealing with FCP involves facing existential questions about the meaning and purpose of life. Spiritual well-being becomes an important coping mechanism in this situation, offering a way to understand suffering, find meaning in adversity, and cultivate inner peace (Butow et al., 2021). Spiritual beliefs can take various forms, including organized religions, personal philosophies, or a connection to nature and the universe, providing a broader context beyond immediate health concerns (Dinkel and Herschbach, 2018). Research has indicated that individuals with strong spiritual well-being may experience reduced levels of anxiety and fear related to cancer progression (Ali et al., 2023; Anderson, 2012). The spiritual aspect offers a unique perspective on the idea of control, allowing individuals to let go of some of the anxiety associated with the unpredictable nature of cancer (Crist and Grunfeld, 2013).

Prior research includes a study on Greek cancer patients that showed a link between higher levels of spiritual well-being and lower FCP (Londoudi et al., 2024). Another review study suggested that psycho-spiritual well-being in advanced cancer patients plays a role in reducing FCP, a key component of psychological distress (Lin and Bauer-Wu, 2003).

In the Iranian context, the link between spiritual well-being and FCP is significant due to the cultural and religious importance of spirituality. Spiritual well-being can play a crucial role in coping with cancer, providing emotional comfort and a sense of meaning in the face of challenges (Ahmadi et al., 2021). However, the specific relationship between spiritual well-being and FCP is not well understood, particularly in the context of Iranian culture, where spiritual beliefs and practices are deeply rooted in everyday life. Recognizing this connection is important for developing culturally appropriate strategies to address FCP, ultimately improving patient care and support (Mardani et al., 2023).

In Iran, spiritual well-being is then profoundly shaped by a rich culture and religious heritage, where Islam holds the upper hand and guides daily life and coping manners. Religious practices among Iranian patients-such as praying, recitation of the Quran, and consulting the religious leader-are very frequent, offering emotional comfort and possibly enhancing perceived control when illness is confronted (Mardani et al., 2023). The cultural background emphasizes community support and shared spiritual values that enhance resilience and point toward a different model of dealing with fear and uncertainty. Understanding these cultural nuances is necessary to make full sense of the way in which spiritual well-being informs coping strategies in Iranian patients with cancer and calls for culturally adapted interventions (Ahmadi et al., 2021).

There is a research gap in the limited studies that specifically examine the cultural dynamics of Iran, where spirituality could potentially help mitigate the psychological effects of FCP (Ahmadi et al., 2021). Closing this gap could offer important information for healthcare providers, allowing them to develop interventions that align with the spiritual and cultural beliefs of Iranian cancer patients, ultimately improving their mental health and quality of life. Therefore, this study sought to explore the intricate connection between spiritual well-being and FCP in individuals facing a cancer diagnosis.

## Materials and methods

### Research design

This study employed a predictive cross-sectional survey design to explore the relationship between spiritual well-being and FCP in cancer patients in Tehran City, Iran.

### Participants

The study included patients who were receiving chemotherapy, radiotherapy, or surgical treatment for cancer, were 18 years or older, and were proficient in reading and writing in Persian. Individuals with psychiatric illnesses were excluded due to the potential confounding effects of these conditions on psychological outcomes, such as anxiety or depression, which could interfere with the study’s focus on spiritual well-being. Similarly, patients with chronic medical conditions unrelated to cancer were excluded to minimize variability in health-related quality of life factors that might skew the results. Informed consent was obtained from all participants prior to the study.

A sample size of 376 was determined using the sample size formula for structural equation modeling with G-Power software (Westland, 2010). This calculation took into account an expected effect size of 0.2, a desired statistical power of 0.8, five latent variables, 40 observed variables (from all of the scales), and a significance level of 0.05. To address potential missing data, the study employed a listwise deletion approach, whereby participants with incomplete responses were excluded from the final analysis. This method was chosen to maintain the integrity of the dataset and ensure robust statistical results (Pepinsky, 2018). The initial recruitment of 398 patients accounted for this possibility, ensuring that the final sample size remained sufficient for reliable analysis and meaningful conclusions. Participants were recruited through convenience sampling from February to May 2023 at two leading comprehensive cancer hospitals (Imam Khomeini and Bu Ali) in Tehran, Iran. All participants completed the scale successfully.

### Measures

#### Spiritual well-being

To assess spiritual well-being, this study utilized the Iranian version of the Spiritual Well-Being Scale (SWBS) (Soleimani et al., 2017). The SWBS consisted of a 10-item religious well-being subscale, which focused on one’s relationship with God, and a 7-item existential well-being subscale, which examined one’s sense of life purpose and life satisfaction. Religious well-being reflects an individual’s relationship with a higher power, offering a sense of divine connection and faith, which can provide solace and strength during illness (Soleimani et al., 2017). For cancer patients, this dimension may help alleviate feelings of helplessness and promote hope through trust in a higher power. Existential well-being, on the other hand, pertains to a sense of meaning and purpose in life, addressing broader existential concerns often intensified by a cancer diagnosis. This dimension allows patients to find significance in their experiences and fosters resilience by reframing suffering as part of a meaningful journey (Sharif Nia et al., 2022).

Participants rated their responses on a 6-point Likert scale ranging from 1 (strongly disagree) to 6 (strongly agree). Scores for each subscale ranged from 7 to 60, with higher scores indicating greater religious or existential well-being. The Persian version of the SWBS has been shown to be reliable and valid for assessing the spiritual well-being of cancer patients (Sharif Nia et al., 2022). The psychometric properties of the SWBS have been evaluated in the Iranian population (Sharif-Nia et al., 2023; Sharif Nia et al., 2018; Soleimani et al., 2017). The reliability of the scale was 0.793 using Cronbach’s alpha.

#### Fear of progression (FOP)

To evaluate the FCP, this study utilized the 12-item FOP Questionnaire (Hinz et al., 2015). Participants provided ratings for each item, such as “Being nervous prior to doctor’s appointment or periodic examinations,” using a 5-point Likert scale ranging from 1 (never) to 5 (very often). The resulting sum score of FoP-Q-12 ranged from 12 to 60. The threshold for dysfunctional Fear of Cancer Progression (FCP) was set at a score of ≥34 on the FOP-Q-12 scale, based on established psychometric guidelines (Hasannezhad Reskati et al., 2022). This cutoff indicates a clinically significant level of fear that may interfere with daily functioning and psychological well-being. Incorporating this threshold provided a clear benchmark for identifying patients requiring targeted psychosocial interventions, ensuring the study’s findings are both clinically meaningful and actionable (Hasannezhad Reskati et al., 2022). The Persian version of the FOP demonstrated satisfactory reliability and validity in patients in Iran (Hasannezhad Reskati et al., 2022). The reliability of the scale was 0.956 using Cronbach’s alpha.

### Data analysis

The data were analyzed using the Statistical Package for Social Sciences version 26.0 software for Windows (IBM SPSS Statistics for Windows, Version 26.0. Armonk, NY: IBM Corp., USA). To assess normal distribution, Kolmogorov–Smirnov tests were employed for continuous variables. Results were presented as mean (SD) and median (Min-Max) for continuous variables, while numbers (percentages) were used for categorical variables.

Confirmatory Factor Analysis (CFA) was conducted on the polychoric correlation matrix using AMOS version 26.0 to validate the internal structure of the constructs. Various goodness-of-fit indices, including the Chi-square statistic (χ2), comparative fit index (CFI), Tucker-Lewis index (TLI), root mean square error of approximation (RMSEA), and standardized root mean square residual (SRMR), were employed to evaluate the fit of the constructs.

In accordance with established criteria (Hu and Bentler, 1999; Marôco, 2021), an acceptable model fit was indicated by CFI and TLI values greater than 0.90, and RMSEA and SRMR values less than 0.06 and 0.08, respectively. For assessing the reliability of the measures, internal consistency analyses were conducted using JASP version 0.18. Specifically, Cronbach’s alpha coefficient (*α*) (Cronbach, 1951), coefficient omega (*ω*) (McDonald, 2013) were computed for each factor. Simple linear regression was employed to analyze the relationship between spiritual well-being and FCP. The significance level for all tests was set at α < 0.05.

Before conducting regression analyses, the assumptions of linearity, multicollinearity, and normality were tested to ensure the validity of the statistical methods. Linearity was confirmed through scatterplots, multicollinearity was assessed using variance inflation factors (VIFs) with acceptable thresholds, and normality was evaluated using the Kolmogorov–Smirnov test. These steps enhanced the reliability of the findings and ensured that the analysis met standard statistical requirements.

### Ethical approval

The Ethical Committee of Mazandaran University of Medical Sciences approved this study (ethics code: IR.MAZUMS.REC.1402.478). All participants signed written consent forms (in printed format) and were assured of privacy. Privacy and confidentiality were strictly maintained by anonymizing data and securely storing all information. Personal identifiers were replaced with unique codes to ensure data confidentiality. They were informed that their participation was voluntary and that they could withdraw from the study at any time.

## Results

The average age of the participants was 49.14 years (standard deviation = 16.16, 95% confidence interval: 47.55, 50.74). Most of the participants were male (56.8%, *N* = 226), and a considerable number (60.6%, *N* = 241) had stage 3 cancer. More information about the demographic characteristics of the patients can be found in Table 1.

**Table 1:** Demographic characteristics of the patients in the study.

Variables	*N* (%)
Sex	
Male	226 (56.8%)
Female	172 (43.2%)
Job	
Housekeeper	94 (23.6%)
Employee	106 (26.6%)
Free lance	107 (26.9%)
Retirement	86 (21.6%)
Other	5 (1.3%)
Marital status	
Single	57 (14.3%)
Married	328 (82.4%)
Divorced	2 (0.5%)
Widow	11 (2.8%)
Educational level	
Elementary	78 (19.6%)
Post elementary	36 (9%)
High school	44 (11.1%)
Diploma	63 (15.8%)
Bachelor	128 (32.2%)
Master and upper	49 (12.3%)
Economic status	
Weak	76 (19.1%)
Average	198 (49.7%)
Good	124 (31.2%)
Cancer stage	
1	5 (%)
2	109 (27.4%)
3	241 (60.6%)
4	33 (8.3%)
Not know	10 (2.5%)

The goodness-of-fit indices and reliability measures for the different constructs, as described in the Methods section, are presented in Table 1. In general, all the constructs showed strong evidence of both factorial validity and reliability, ensuring solid validity and reliability (Table 2).

**Table 2:** Goodness of fit indices and reliability measures for the variables used in the analysis.

Construct	Factor’s loadings range	Fit indices	Reliability measures**
Spiritual well-being - Believe in God* - Confusion about God*	0.663–0.834 0.526–0.673	CFI = 0.834 TLI = 0.812 SRMR = 0.168 RMSEA = 0.13	ω_t_ = 0.689 *α* = 0.934; *ω* = 0.933 *α* = 0.934; *ω* = 0.933
FCP	0.724–0.891	CFI = 0.918 TLI = 0.981 SRMR = 0.124 RMSEA = 0.112	*α* = 0.956; *ω* = 0.957

*Latent variables of spiritual well-being; **ω, McDonald’s omega; α, Cronbach’s alpha; FCP, Fear of cancer progression.

The data was found to be normally distributed based on the Kolmogorov–Smirnov test (*p* > 0.05). The average score for spiritual well-being was 48.89 (SD = 9.40, 95% CI: 47.96, 49.82). The mean scores for religious well-being and existential well-being were 50.42 (SD = 7.89) and 32.78 (SD = 5.11) respectively. The average FCP score was 48.89 (SD = 13.62, 95% CI: 43.45, 46.14).

Table 3 displays the results of the simple linear regression analysis, indicating that spiritual well-being significantly predicted FCP (*R*^2^ = 0.064, *F* = 27, *p* < 0.001). Furthermore, the multiple linear regression analysis demonstrated a significant association between economic status and FCP (*R*^2^ = 0.12, *F* = 54.03, *p* < 0.001).

**Table 3:** Results of fear of cancer progression predictor variables.

Predictive variables	Simple linear regression				
	B	β	*t*-value	*p*-value	CI 95%
Spiritual well-being	0.366	0.253	5.19	<0.001	0.227 to 0.504
	Multiple linear regression				
Age, (year)	0.085	0.101	1.906	0.057	−0.003 to 0.174
Sex, (F/M)	−0.329	−0.012	−0.26	0.795	−2.82 to 2.16
Educational level	−0.672	−0.085	−1.57	0.11	−1.51 to −0.16
Economic status	6.69	0.34	7	<0.001	4.81 to 8.56
Cancer stage	0.94	0.04	1.04	0.29	−0.83 to 2.73

B, Unstandardized Coefficients; β, Standardized Coefficient.

## Discussion

The study’s findings indicated that spiritual well-being directly predicts FCP. Scholars globally have determined that religion and spirituality play a crucial role in FCP (Ali et al., 2023; Butow et al., 2021; Lim et al., 2022; Niu et al., 2019). Cancer, with its unpredictable nature and potential for advancement, frequently prompts individuals to contemplate existential questions and delve into the meaning of life. Spiritual well-being acts as a valuable coping strategy, equipping individuals with tools to manage the emotional challenges associated with FCP (Ellington et al., 2017).

Londoudi et al. (2024) found that higher levels of spiritual well-being were associated with lower levels of fear of cancer recurrence, which aligns with the results of our study. Previous research has consistently shown a positive relationship between spiritual well-being and both physical and mental health (Albusoul et al., 2022; Zare et al., 2019). Improved spirituality has been linked to better adaptation to difficult life events and more effective coping strategies (Azar et al., 2022). A randomized controlled trial by Sajadian et al. (2021) showed that transpersonal therapy, which includes spiritual therapy and yoga meditation, significantly reduced fear of cancer recurrence in breast cancer survivors. Another study found that patients engaged in various spiritual practices as a way to cope with and reduce their fear of recurrence (Ali et al., 2023).

With spiritual wellbeing, although statistically contributing to FCP, it had an R-squared value of 0.064, which is very small. The implication is that spiritual wellbeing is important, but at the same time, other psychosocial, medical, or contextual variables may be playing major roles in shaping the experiences of FCP (Zhang et al., 2022). It has implications for clinical practice since it gives notice on the added value of integrating spiritual wellbeing into a broader multidisciplinary approach for dealing with FCP. Spiritual care may then be provided in a targeted manner to support other therapeutic approaches, reinforcing one another in offering holistic support to the patient, even when its direct effect on FCP is limited.

Existing literature indicates that spirituality is more closely linked to psychological well-being than religiosity (Fradelos et al., 2021). In a study by Nelson on prostate cancer patients, the relationship between spirituality, religiosity, and depression was examined (Nelson et al., 2009). The study hypothesized that spirituality plays a mediating role in the connection between religiosity and depressive symptoms. Results showed that strong religious beliefs were effective in reducing depressive symptoms only for individuals who derived meaning from their religion. Spirituality and psychological resilience are crucial for managing challenging life circumstances, especially in alleviating concerns about cancer progression.

Spirituality can provide individuals with a sense of inner strength and control, helping them tap into reserves of resilience during uncertain times. Belief in a higher power or greater purpose can empower individuals to confront their fears with a perspective that goes beyond immediate circumstances (Mardani et al., 2023). Dealing with FCP can be a lonely journey, causing individuals to question the meaning and purpose of their lives. Spiritual beliefs offer a way to identify purposes in the face of adversity (Alvarenga et al., 2021). Whether through a connection to a divine plan, a commitment to personal growth, or a sense of contributing to a larger good, spirituality allows individuals to reframe their story and find meaning even in the midst of medical challenges (Ali et al., 2023).

Many spiritual practices emphasize mindfulness and are currently prevalent. Whether through prayer, meditation, or other contemplative exercises, individuals can cultivate awareness of the present, shifting their focus from future uncertainties to their immediate experiences (Park et al., 2020). This mindfulness not only helps reduce anxiety about potential cancer progression but also fosters a deeper appreciation for life as it is now. Spiritual well-being encompasses a set of beliefs that often include ideas of purpose, interconnectedness, and transcendence (Park et al., 2020). These beliefs serve as sources of emotional resilience, providing a broader perspective that goes beyond the immediate challenges of illness (Zhang et al., 2022). Trust in a higher power or belief in the transformative nature of suffering can strengthen emotional resilience, helping individuals navigate the emotional highs and lows of their cancer journey.

Spiritual well-being involves personal beliefs and practices and often includes a communal aspect, which can provide a supportive network that has a profound impact on individuals dealing with FCP (Ban et al., 2021). This community connection is essential in offering emotional, practical, and spiritual support, contributing to a more holistic approach to dealing with the challenges of illness. Being part of a spiritual community involves sharing common beliefs, values, and perspectives (Hauken and Larsen, 2019), which creates a special bond among individuals facing FCP within the same community. Knowing that others in the community can relate to the spiritual and existential aspects of the journey brings comfort and fosters a sense of unity and shared strength (Yang et al., 2018).

Spiritual communities often function as support systems where individuals can openly share their fears, doubts, and hopes in a non-judgmental setting. The empathy and understanding found within these communities create a safe environment for emotional expression, reducing the sense of isolation that can come with dealing with a potentially progressive illness (Liu et al., 2022). In addition to emotional support, spiritual communities often offer practical assistance and compassionate care. Whether through support groups, outreach programs, or individual acts of kindness, members of these communities may provide tangible help such as transportation to medical appointments, meal support, or simply being there for someone in need (Reb et al., 2020). Spiritual communities also frequently participate in collective healing and prayer rituals, which serve as a shared expression of hope and create a collective energy believed to positively impact the well-being of those facing illness. These rituals promote a sense of interconnectedness and shared responsibility for each other’s well-being (Bergerot et al., 2022).

The spiritual well-being of Iranian cancer patients is deeply influenced by Islamic practices and beliefs, which serve as vital coping mechanisms. Practices such as prayer, Quran recitation, and reliance on divine wisdom (Tawakkul) provide emotional solace and resilience (Khiyali et al., 2023). Islamic teachings, which often frame suffering as a test of faith or spiritual growth, may help reframe the cancer experience positively, reducing FCP. Additionally, the communal aspects of Islam, such as group prayers and support networks, foster a shared sense of strength and hope (Khiyali et al., 2023).

Many spiritual traditions highlight the transformative power of suffering. In this context, the challenges presented by cancer progression are seen as opportunities for personal growth, resilience, and spiritual advancement (Dunn et al., 2015). The idea that adversity can result in positive change instills a sense of hope, prompting individuals to perceive their difficulties as part of a broader journey toward personal and spiritual growth. Spirituality often underscores the interconnectedness of all beings (Mardani et al., 2023). This interconnected view fosters collective resilience, where the optimism and hope of one person contribute to the well-being of the entire community. Feeling connected to a larger network of support boosts individual resilience, as individuals draw strength not only from their personal beliefs but also from the shared hope of the spiritual community (Ellington et al., 2017).

Spiritual well-being often involves having faith in the potential for healing, whether through medical treatment, alternative therapy, or divine intervention. This faith serves as a source of hope and optimism, shaping individuals’ attitudes toward their health. Believing in the possibility of recovery, even in the midst of cancer progression, fosters a resilient mindset that can have a positive impact on the course of illness (Pradhan et al., 2021). Spiritual teachings often include positive affirmations and guidance on maintaining a hopeful and optimistic outlook. Scriptures, sacred texts, or teachings from spiritual leaders may provide words of encouragement, highlighting the importance of maintaining hope in difficult times. Individuals often draw inspiration from these affirmations, which help fuel their resilience (Seiler and Jenewein, 2019).

The multiple regression analysis also identified economic status as a significant predictor of FCP, underscoring the role of financial stress in shaping patients’ psychological experiences. Financial difficulties can exacerbate fears about the progression of illness, particularly in contexts where treatment costs are high or insurance coverage is limited (Yang et al., 2018). This stress may interact with spiritual well-being by intensifying existential concerns or reducing the time and energy available for spiritual practices. Patients burdened by economic challenges may find it more difficult to focus on prayer or engage in community support, both of which are critical aspects of spiritual well-being (Niu et al., 2019).

### Limitations and strength

The study focused on cancer patients in Tehran City (Tehran, Iran), which may limit the generalizability of the findings to other cultural or ethnic groups. Cultural factors can significantly influence spiritual well-being and FCP, but these factors may not be universally applicable. The relatively small effect size observed in the regression analysis suggests that spiritual well-being, while significant, is not the sole factor influencing FCP. Other unmeasured variables, such as personality traits or family dynamics, may also play a role and warrant further investigation. This study relied heavily on self-report measures for assessing spiritual well-being and FCP, and there is a risk of response bias and social desirability.

Furthermore, this study delves into the connection between spiritual well-being and FCP, shedding light on a pertinent issue in clinical practice. The results have the potential to inform interventions designed to enhance the mental well-being of cancer patients. By specifically examining the Iranian cultural context, this research may reveal cultural intricacies that impact the correlation between spiritual well-being and FCP, thereby enriching the worldwide comprehension of this intricate topic.

### Clinical implications

To enhance the spiritual well-being of cancer patients, healthcare providers should integrate spiritual care into standard psychosocial interventions. By incorporating culturally sensitive spiritual support, such as guided religious practices, spiritual counseling, or collaboration with religious advisors, healthcare providers can address both the emotional and existential challenges faced by patients. These findings underscore the importance of a multidisciplinary approach that values spiritual care as a key component of comprehensive cancer management, ultimately enhancing patient resilience and quality of life.

Partnering with Islamic scholars or chaplains familiar with patients’ cultural and religious contexts to provide tailored spiritual guidance. This could involve facilitating prayer sessions, Quranic recitations, or individual counseling. Designing interventions such as mindfulness meditation grounded in Islamic teachings, group discussions on the spiritual meaning of illness, or workshops focusing on finding purpose through adversity.

Establishing interdisciplinary teams, including spiritual advisors alongside psychologists and medical staff, to address patients’ holistic needs comprehensively. Creating peer-led groups that emphasize shared religious and spiritual practices to build community and collective resilience. Training healthcare professionals to recognize spiritual distress and collaborate effectively with spiritual advisors, enhancing their ability to support patients’ spiritual well-being.

## Conclusion

The results of our research emphasize the important connection between spiritual well-being and fear of cancer recurrence (FCP) in cancer patients. Increased spiritual well-being was linked to decreased FCP levels, indicating that spirituality plays a crucial role in helping patients cope with the emotional challenges related to fears of cancer returning. These findings underscore the significance of incorporating spiritual support into cancer treatment plans to address the psychological and emotional well-being of patients.

## Data Availability

The raw data supporting the conclusions of this article will be made available by the authors, without undue reservation.
